The article "Clinical Effects of Acupuncture for Stroke Patients Recovery" was retracted in 2023. Reasons: signs of a paper mill; compromised peer review; unreliable results or conclusions.

# Clinical Effects of Acupuncture for Stroke Patients Recovery

**DOI:** 10.1155/2022/9962421

**Published:** 2022-02-14

**Authors:** Xia Guo, Bingjie Cheng

**Affiliations:** ^1^Rehabilitation Department of Traditional Chinese Medicine, Hanyang Hospital of Wuhan University of Science and Technology, Wuhan 430050, China; ^2^Traditional Chinese Medicine Department, Hubei No. 3 People's Hospital of Jianghan University, Wuhan 430033, China

## Abstract

Stroke is assumed as one of the common cerebrovascular diseases that endangers human health and life. Its incidence and mortality rates are high, while survivors (50% to 70%) suffer from different degrees of disability. Hemiplegia is a common disability after stroke, mainly manifested as muscle weakness of the affected side, limb spasm, and limited activity, which severely impacts a patient's daily life. There are various rehabilitation methods for stroke hemiplegia, including modern rehabilitation medicine, motor therapy, acupuncture, and rehabilitation robot. The cost and effect of different rehabilitation methods are not the same. It is the focus to find an economical and effective rehabilitation method. In this paper, 128 stroke patients aged 41 to 73 hospitalized between January 2019 and January 2021 were analyzed. The intervention group used standard physical therapy and traditional acupuncture therapy, and the control group only used standard physical therapy. We used RStudio 1.1.419 (RStudio Corporation) for analysis. Experimental results show that the short-term efficacy of the intervention group is better than that of the control group. The intervention group was better than the control group in recovery from injury during rehabilitation, degree of muscle spasm, self-care ability in daily life, and overall degree of damage. In the long-term efficacy analysis, we can see that with the increase in the number of acupuncture, the efficacy of the intervention group is still better than that of the control group. Compared with physical rehabilitation alone, acupuncture has better short-term, and long-term clinical effects for stroke patients improves motor dysfunction and improves the quality of life and independence of stroke patients. With the increase in the number of acupuncture treatments, the patient's rehabilitation effect will be better.

## 1. Introduction

Stroke is the first disability disease in the world in the past ten years [1]. With the aging population, the incidence rate of stroke is increasing, causing pain to patients and bringing a severe burden to society and families [2]. Rehabilitation treatment after stroke is a complex and lengthy process, which requires a large amount of human and financial input [3]. Some stroke patients in underdeveloped areas stop thinking that treatment is essential and rehabilitation is not crucial. Because of the lack of regular rehabilitation training, the patients miss the best recovery time, which is prone to residual muscle contracture, joint deformity, and other sequelae [4]. Some studies have shown that the brain has certain plasticity and can be used for functional reorganization [5]. After a stroke, the injured nervous system can be adapted to the external stimulation, and the damaged nerve tissue can play a compensatory role. The damaged nerve cells can grow axons and dendrites again, which is beneficial to reconstructing the neural pathway. Therefore, the training stimulation can promote the reconstruction and recovery of nerve function [6]. At the same time, the study holds that rehabilitation treatment of cerebrovascular diseases should not be limited to some treatment methods but should be combined with various rehabilitation treatment methods according to the actual situation [7].

The article "Clinical Effects of Acupuncture for Stroke Patients Recovery" was retracted in 2023. Reasons: signs of a paper mill; compromised peer review; unreliable results or conclusions.

Rehabilitation training is the primary way to promote the recovery of limb function in stroke patients with hemiplegia [8]. Some neurophysiologists supported that standardized rehabilitation training stimulation can promote nerve cell protrusion near the lesion, accelerate the proliferation of peripheral glial cells and vascular endothelial cells, which is conducive to the repair of the lesion [9]. Rehabilitation training can promote the compensation and reorganization of intact nerve cells and accelerate new neural pathways [10]. Rehabilitation training can also regulate the highest peripheral, central function by enhancing the input stimulation of the infarcted cortex, which is conducive to enhancing brain plasticity, promoting the recovery of limb motor function and improving patients' self-care ability [11]. From the perspective of motor function, rehabilitation training enables patients to participate in limb movement and daily activities, which can strengthen muscle and joint activities, improve patients' muscle strength, and facilitate the recovery of related functions and daily activities [12]. Acupuncture, originated from traditional Chinese medicine, has a low cost, and the World Health Organization has recognized its effect in the rehabilitation of brain injury-related diseases [13]. It has been proved that acupuncture can dilate blood vessels, improve cerebral circulation, improve blood oxygen supply of damaged nerve tissue, and reduce the generation of free radicals [14]. Acupuncture is conducive to neuron protection, prominent formation, and neural stem cell proliferation. Also, acupuncture promotes the repair of nerve function [15].

The article "Clinical Effects of Acupuncture for Stroke Patients Recovery" was retracted in 2023. Reasons: signs of a paper mill; compromised peer review; unreliable results or conclusions.

Some studies have confirmed that acupuncture can improve motor dysfunction, quality of life, and independence of stroke patients [6, 12]. However, in recent years, some studies have some limitations that the clinical trial design of acupuncture in treating stroke patients with dyskinesia is unreasonable. There are no controlled randomized controlled trials, and there is a lack of large sample size experimental studies. Some studies even show that acupuncture does not affect acute stroke. Therefore, we conducted this research to analyze acupuncture in stroke recovery in the short and long term.

In this paper, 128 stroke patients aged 41 to 73 hospitalized between January 2019 and January 2021 were analyzed. The intervention group used standard physical therapy and traditional acupuncture therapy, and the control group only used standard physical therapy. We used RStudio 1.1.419 (RStudio Corporation) for analysis. Experimental results show that the short-term efficacy of the intervention group is better than that of the control group. The intervention group was better than the control group in recovery from injury during rehabilitation, degree of muscle spasm, self-care ability in daily life, and overall degree of damage. In the long-term efficacy analysis, we can see that with the increase in the number of acupuncture, the efficacy of the intervention group is still better than that of the control group.

The rest of the manuscript is arranged accordingly as follows.

In Section 2, the proposed method is defined and presented in an easy way to enable various readers to understand it easily. In Section 3, the proposed scheme is implemented in a real environment; hence, various results were described and presented with complete analysis along with the supported literature review or methods which are already available. A generalized discussion section is provided in Section 4 where the problem under consideration is defined along with the proposed solution and its effectiveness. Finally, concluding remarks are provided along with the references which are used in the article.

## 2. Proposed Methodology and Materials

### 2.1. Patients

In this study, 128 stroke patients aged 41 to 73 years hospitalized between January 2019 and January 2021 were analyzed.

The inclusion criteria were as follows:

1. Patient was diagnosed by CT or MRI and met the diagnostic criteria of “diagnostic points of various cerebrovascular diseases [6]”
2. The Patient's condition was stable
3. Patients were in the recovery period
4. Patients had hemiplegic manifestations such as unilateral muscle weakness and limb spasm
5. Patients had no apparent cognitive impairment
6. Patients had good treatment compliance

Exclusion criteria for patients were as follows:

1. Brain trauma
2. Cerebral hemangioma
3. Organ dysfunction
4. Other severe diseases due to joint deformity, rheumatism, and other sports disorders
5. Mental illness, cognitive impairment, and poor treatment compliance

The article "Clinical Effects of Acupuncture for Stroke Patients Recovery" was retracted in 2023. Reasons: signs of a paper mill; compromised peer review; unreliable results or conclusions.

### 2.2. Study Design

The study was a retrospective case-control study with a blind evaluator method, involving two groups: the intervention group received standard physical therapy and traditional acupuncture while the control group only received standard physical therapy. The physiotherapists recorded the patients' demographic data and functional status during patients receiving treatment. Therefore, physiotherapists do not know whether patients are receiving acupuncture intervention outside of their daily work. We analyzed the data anonymously, and the review committee approved the exemption of informed consent.

### 2.3. Outcome Assessment

This study used the Fugl–Meyer scale, modified Ashworth scale, Barthel index, and NIH Stroke Scale as the primary outcome measures. Taking the Kaplan–Meier curve of acupuncture frequency and stroke improvement as the secondary result, we compared the acupuncture and control groups from multiple perspectives.

### 2.4. Intervention

Patients in two groups received conventional drugs during the rehabilitation treatment. The control group received comprehensive rehabilitation training. The training was based on the recovery stage of hemiplegia to formulate the targeted rehabilitation objectives and training contents. During the soft paralysis period, the leading training contents prevent joint contracture, improve regular sensory motor stimulation, induce active exercise, and avoid complications and secondary injury. The training contents include

1. Turning over the bed, 4 hours/time
2. Good limb position
3. Breathing training
4. Joint passive activity training
5. Muscle strength training
6. Sitting and balance training and
7. Standing training

During the period of spasticity, the leading training contents are to reduce muscle tension, improve spasticity mode, and improve separation movement;

1. Body position conversion
2. Trunk muscle stretching
3. Standing balance
4. Gait training
5. Transfer of gravity center
6. Pelvic separation training in sitting position
7. Speech and swallowing training

During the recovery period, the patients' activities of daily living were mainly improved, including

1. Walking training
2. Up and downstairs training
3. Limb coordination training
4. Daily activities training such as transfer, dressing, eating, and toilet

The training was given once a day, 45 min to 1 h for each training, 5-6 days a week. The intensity is suitable for patients without apparent fatigue. Family members can train to ensure the training intensity and quality—continuous training for eight weeks during the training period.

The article "Clinical Effects of Acupuncture for Stroke Patients Recovery" was retracted in 2023. Reasons: signs of a paper mill; compromised peer review; unreliable results or conclusions.

The intervention group received acupuncture treatment on top of the control group, and the diameter of the selected scalp needle is 0.3 mm, body acupuncture 0.25 mm × 40 mm, and waist-hip 0.25 mm × 75 mm. According to Brunnstrom stage of hemiplegia [12], in Brunnstrom stage I-II (mild paralysis stage), Neiguan, Sanyinjiao, and Shuigou were selected as the main points; Chize, Jiquan, and Weizhong on the affected side were selected as the auxiliary points; Yanglingquan, Zusanli, and Futu were selected as the matching points; and the oblique needling depth was 0.5–1.0 inch (1.67–3.33 cm). In Brunnstrom stage III-IV (spasmodic stage), we selected the upper limbs from Tianjing, Yangchi, Jianzhen, Gai, Zhongzhu, Shousanli, Yangguan, and other acupoints on the affected side, and we chose the lower limbs from Weizhong, Weiyang, Yinmen, Yanglingquan, Zhaohai, Chengshan, and different acupoints, 2-3 points each time to avoid muscle spasm after acupuncture. In Brunnstrom stage V-VI (recovery stage), based on the spasmodic stage, acupuncture at Zusanli, Shousanli, Sanyinjiao, and other acupoints were added.

### 2.5. Statistical Analysis

Data collection follows the requirements of retrospective research. Both the baseline data and the result data are descriptive studies, and differences are analyzed. The average ± SD determines continuous variable data, and discontinuous variables are displayed as counts. RStudio 1.1.419 (RStudio Inc) was used for statistical analysis. Student's *t*-test was used for continuous variables, and Kruskal–Wallis test or Mann–Whitney test was used for nonparametric variables. The chi-square test and Fisher's precision test were utilized for discontinuous variables. *P* < 0.05 is statistically significant.

## 3. Experimental Results

In this section, a brief but comprehensive comparative study of the proposed study in terms of the experimental results and observations is presented.

### 3.1. Patient Characteristics

We included one hundred twenty-eight subjects in this study, of which 65 were in the intervention group and received acupuncture plus physical therapy. In contrast, 63 in the control group received only physical therapy. From the comparison of baseline data, we can see no difference in age, gender, BMI, length of stay, hypertension, and intervention interval between the two groups, which is comparable, as given in Table 1.

In Table 2, we list the clinical efficacy and scores of the two groups. The difference in the total effective rate between the two groups is statistically significant, and the intervention group is higher than the control group. Fugl–Meyer Assessment (FMA) scale is an index to assess the sensorimotor impairment in individuals who had a stroke. The results showed that FMA in the intervention group was higher than that in the control group, indicating that the motor function of the intervention group was better than that of the control group. The modified Ashworth scale is a muscle tone assessment scale used to assess the resistance experienced during passive range of motion. The increase of muscle tension in the intervention group was lower than that in the control group. The Barthel scale/index (BI) is an ordinal scale used to measure performance in activities of daily living (ADL). The NIH Stroke Scale (NIHSS) is a standardized scoring tool used by physiologists and other healthcare professionals to measure and record the level of injury caused by a stroke.

The article "Clinical Effects of Acupuncture for Stroke Patients Recovery" was retracted in 2023. Reasons: signs of a paper mill; compromised peer review; unreliable results or conclusions.

Finally, we made the Kaplan–Meier survival curve of stroke improvement, with the number of acupuncture accepted as the abscissa and the practical improvement of stroke as the ordinate. We can see from Figure 1 that compared with the control group, the functional improvement of stroke gradually increases with the times of acupuncture incline. The difference between the two groups had significance and intervention is better than the control group.

## 4. Discussion

This study shows that the intervention group is better than the control group in short-term efficiency. The intervention group was better than the control group in the scales, including the recovery of injury during rehabilitation, the degree of muscle spasm, self-care of daily life, and the overall degree of damage. In the analysis of long-term efficacy, we can see that the effectiveness of the intervention group is still better than that of the control group with the increase in the number of acupuncture treatments. In conclusion, acupuncture has better short-term and long-term effects on the rehabilitation of stroke patients on the premise of comparability between the two groups.

The mechanism of acupuncture improving stroke may include the following aspects: the cascade reaction of ischemic stroke involves a variety of essential processes. Acupuncture is involved in multiple interventions in the cascade reaction from the beginning to the end of the stroke, such as cell damage caused by hypoxia and glucose deficiency at the beginning of the stroke, and then affects a variety of interdependent molecular pathways, including excitotoxicity, acidosis, hyperglycemia ion imbalance, and inflammation [16]. To improve the blood flow in the ischemic area of the brain, the high metabolic activity of the brain depends on the continuous supply of oxygen and glucose in the blood circulation [17]. In contrast, the storage level of energy and metabolites of the brain itself is shallow, which means that the brain is vulnerable to blood flow interference [18]. Some studies have found that acupuncture for early stroke (12–24 h) can promote the expression of vascular endothelial growth factor (VEGF), which helps to restore oxygen or nutrition supply in the ischemic penumbra [19]. Acupuncture also provides a beneficial environment for injured tissue, providing a theoretical basis for acupuncture intervention in early stroke [20]. In the acute phase of ischemia, vasodilator mediators (such as nitric oxide) are the key to reduce infarct focus and related secondary damage [21]. Baldo et al. reported that acupuncture could regulate vasoactive substances and activate nitric oxide synthase III, and it also inhibits the angiotensin system and platelet adhesion. Inflammatory response after cerebral ischemia is mainly mediated by microglia, astrocytes, and leukocytes, including cytokines (IL-1, IL-6, IL-10, and TNF-*α*) [22]. This inflammatory response induces the activation of gene expression and transcription factors that regulate the ischemic cascade and further aggravates the local inflammatory response. Pinedo et al. reported that acupuncture at Zusanli, Baihui, and Quchi could significantly improve the local anti-inflammatory effect of ischemic stroke in rats [14]. They believed that acupuncture could improve the local anti-inflammatory effect of ischemic stroke by inhibiting local inflammatory factors (including TNF-*α*), heat shock protein 70 (HSP70), and toll-like receptor (TLR) released to control the inflammatory process [23].

The article "Clinical Effects of Acupuncture for Stroke Patients Recovery" was retracted in 2023. Reasons: signs of a paper mill; compromised peer review; unreliable results or conclusions.

Acupuncture promotes the formation of the central nervous system and cell proliferation and enhances serine protein kinase/protein phosphatase 2 (GSK-3 *β*/PP2A) expression [16]. GSK-3 *β*/PP2A is a group of biological proteins related to phosphorylation and cell proliferation. The balance of protein activity and its presentation are closely related to the control of central nervous system neurons [24]. In addition, acupuncture can increase brain-derived neurotrophic factors (BDNFs) and VEGF. BDNF/VEGF, as an essential nutrient medium for neural stem cells, can stimulate the growth of new nerves and the migration of neural source areas [25]. Huili and Wu reported that acupuncture was beneficial to stem cell differentiation after cerebral ischemia, increased BDNF and VEGF, and upregulated neuroprotective substances [9]. Acupuncture can also promote the proliferation of cells in ischemic damaged tissues. It activates the Wnt/*β*-catenin signal pathway and promotes the proliferation of astrocytes and neural stem cells [26]. In addition, acupuncture also increases cyclin expression by upregulating the expression of stem cell factor, c-kit gene, matrix metalloproteinase nine, and mRNA [27]. Antiapoptosis is one of the most common mechanisms of acupuncture in the treatment of stroke. After a stroke, apoptosis occurred in the neuronal population, and the apoptosis signal level was formed by two apoptosis pathways (endogenous/exogenous) [28]. The endogenous apoptosis in the ischemic region is mediated by caspase-1 and caspase-3, which release cytochrome c from mitochondria by activating the internal apoptosis pathway. Exogenous pathways play a role in the related processes, such as oxygen-free radical release, death receptor, DNA damage, and protease activation. Stimulation of acupoints in Zusanli, Hegu, Qihai, and Xuehai can inhibit apoptosis factors c-fos, caspase-3, and Bax and regulate the expression of the protective protein [29].

Acupuncture can also help to restore the memory and learning process of the hippocampus. Stroke patients often have different degrees of cognitive impairment, among which memory impairment is the most common [30]. The results showed that the glucose metabolism and dopamine level in the hippocampus, amygdala, and caudate putamen increased after electroacupuncture of Baihui and shunting, which reduced brain atrophy and improved the neuron defect [9]. Excessive glutamic acid can damage neurons and induce extemporaneous toxicity. It not only affects the infarcted area but also damages the CA1 subfield of the hippocampus [19]. Chen et al. found that EA could decrease glutamate release in hippocampal CA1 subfield and inhibit hyperemia during reperfusion [6]. Long-term potentiation is an essential cellular model of hippocampal synaptic transmission learning and memory formation. Camp/PKA-CREB is one of the most critical central molecular pathways of long-term memory formation [13].

## 5. Conclusion and Future Study

In this paper, 128 stroke patients aged 41 to 73 hospitalized between January 2019 and January 2021 were analyzed. The intervention group used standard physical therapy and traditional acupuncture therapy, and the control group only used standard physical therapy. We used RStudio 1.1.419 (RStudio Corporation) for analysis. Experimental results show that the short-term efficacy of the intervention group is better than that of the control group. The intervention group was better than the control group in recovery from injury during rehabilitation, degree of muscle spasm, self-care ability in daily life, and overall degree of damage. In the long-term efficacy analysis, we can see that with the increase in the number of acupuncture, the efficacy of the intervention group is still better than that of the control group. Compared with simple physical rehabilitation, acupuncture has a better short-term and long-term clinical effect on stroke patients, improves motor dysfunction, and improves the quality of life and independence of patients with stroke. With the increase of acupuncture treatment times, the rehabilitation effect of patients will be better.

The article "Clinical Effects of Acupuncture for Stroke Patients Recovery" was retracted in 2023. Reasons: signs of a paper mill; compromised peer review; unreliable results or conclusions.

The proposed approach can be an effective mechanism for the physical therapy of elderly patients specifically those with knee injuries.

## Figures and Tables

**Figure 1:** Kaplan–Meier curves of two groups comprised those for whom acupuncture was initiated within 3 months of stroke onset.

**Table 1:** Baseline demographic of two groups.

Variable	Intervention (*n* = 65)	Control (*n* = 63)	*χ* ^2^/*t* value	*P* value
Age (years)	63.25 ± 12.32	64.19 ± 11.21	−0.45	0.65
Gender (male/female)	44/21	43/20	0	1
BMI	25.52 ± 3.12	25.51 ± 3.62	0.02	0.99
Onset duration (d)	36.5 ± 35.8	32.7 ± 37.8	0.58	0.56
Hypertension	56	54	0	1
Intervention period (d)	20.5 ± 7.8	18.1 ± 8.4	1.68	0.09

**Table 2:** Clinical effects after treatment in two groups.

Variable	Intervention (*n* = 65)	Control (*n* = 63)	*χ* ^2^/*t* value	*P* value
No.effective	59	45	6.64	<0.01
Fugl–Meyer scale	66.24 ± 11.85	52.52 ± 9.58	7.19	<0.01
Modified Ashworth scale	2.02 ± 0.48	3.25 ± 1.25	7.31	<0.01
Barthel index	82.25 ± 11.25	69.54 ± 8.65	6.15	<0.01
NIH stroke scale	7.24 ± 5.85	9.52 ± 6.51	−2.09	0.04

## Data Availability

The datasets used and analyzed during the current study are available from the corresponding author upon reasonable request.
